# Histone Lactylation‐Driven Upregulation of VRK1 Expression Promotes Stemness and Proliferation of Glioma Stem Cells

**DOI:** 10.1002/advs.202503897

**Published:** 2025-09-24

**Authors:** Jinna Li, Chenyue Tang, Xuefeng Zhang, Rui Xing, Qing Guo

**Affiliations:** ^1^ Department of Oncology Shengjing Hospital of China Medical University Shenyang Liaoning 110004 China; ^2^ Department of Neurosurgery The First Hospital of China Medical University Shenyang Liaoning 110001 China; ^3^ Institute of Nervous System Diseases Xuzhou Medical University Xuzhou Jiangsu 221002 China

**Keywords:** glioma stem cell, histone lactylation, nanoliposome, SOX2, VRK1

## Abstract

Glioblastoma (GBM) is the most malignant primary brain tumor in adults, with glioma stem cells (GSCs) as a subpopulation contributing to treatment resistance and recurrence. This study investigates the role of lactate and its regulatory gene, vaccinia‐related kinase 1 (*VRK1*), in the regulation of GSC stemness. Utilizing multiple glioma‐related databases and patient‐derived GSCs, it is discovered that lactate enhances the stemness and proliferation of GSCs via VRK1. Mechanistically, lactate promotes histone lactylation (H3K18la) at the *VRK1* promoter in GSCs, thereby upregulating VRK1 expression. VRK1 enhances Y‐box binding protein 1 (YBX1) protein stability by inhibiting its ubiquitination and degradation, and phosphorylates YBX1 to promote its nuclear translocation, thereby regulating GSC stemness and proliferation via the YBX1/SOX2 pathway. Additionally, the VRK1‐targeted nanoliposome A/TMZ‐siVRK1 effectively suppresses the stemness and proliferation of GSCs, demonstrating its therapeutic potential. In conclusion, lactate regulates the stemness and proliferation of GSCs via the H3K18la/VRK1/YBX1/SOX2 pathway. This study elucidates the role of histone lactylation in stem cell regulation and suggests that VRK1 is a potential therapeutic target for GBM.

## Graphical abstract

Glioblastoma (GBM) is the most aggressive primary brain tumor, with glioma stem cells (GSCs) driving treatment resistance. This study reveals that lactate promotes histone lactylation (H3K18la) at the *VRK1* promoter, regulating GSC stemness and proliferation via the H3K18la/VRK1/YBX1/SOX2 pathway. The VRK1‐targeted nanoliposome A/TMZ‐siVRK1 demonstrates therapeutic potential in GBM. These findings underscore the role of histone lactylation in stem cell regulation.

## 1 Introduction

Glioblastoma (GBM) is the most common and aggressive primary malignant tumor of the adult central nervous system.^[^ ^1^ ^]^ Due to its infiltrative growth into surrounding brain tissue, the difficulty of complete surgical resection, and the limited efficacy of radiotherapy and chemotherapy, GBM is characterized by a high recurrence rate and poor prognosis. Current treatment strategies for GBM primarily focus on maximal surgical resection combined with temozolomide (TMZ) chemotherapy and adjuvant radiotherapy. In recent years, molecular targeted therapy and immunotherapy have emerged as additional treatment modalities for GBM; however, the median survival time remains dismally low.^[^ ^2^, ^3^ ^]^ Cancer stem cells (CSCs) are defined as a unique subset of tumor‐initiating cells capable of self‐renewal, multilineage differentiation, high proliferation, and treatment resistance.^[^ ^4^ ^]^ CSCs are more prevalent in highly malignant tumors, such as GBM.^[^ ^5^ ^]^ Glioma stem cells (GSCs) have been identified in GBM and exhibit characteristics such as high aggressiveness, recurrence, angiogenesis, and treatment resistance.^[^ ^6^, ^7^, ^8^ ^]^ Due to their enhanced DNA repair capacity, GSCs can rapidly recover from traditional therapeutic stress, leading to resistance against antitumor treatments such as TMZ.^[^ ^7^, ^8^, ^9^ ^]^ Studies have shown that transcription factors such as SOX2, POU3F2, and OLIG2 can reprogram differentiated glioma cells (DGCs) into stem‐like tumor cells.^[^ ^10^ ^]^ Advances in GSC research have opened new avenues for elucidating the molecular mechanisms underlying the initiation and progression of GBM, as well as for developing novel diagnostic and therapeutic strategies. Targeting GSCs is expected to help overcome the current treatment bottleneck in GBM.

Tumor cells exhibit a unique metabolic pattern in which they do not undergo complete oxidation, even under oxygen‐rich conditions, but instead rely on glycolysis to produce lactate—a phenomenon known as aerobic glycolysis, or the Warburg effect.^[^ ^11^ ^]^ Lactate not only serves as a metabolic substrate for energy production but also functions as a signaling molecule that regulates various tumor‐associated physiological processes, including cell cycle regulation, immune suppression, and energy metabolism alterations.^[^ ^12^ ^]^ Elevated lactate levels are associated with poorer clinical outcomes in multiple tumor types.^[^ ^13^, ^14^, ^15^, ^16^, ^17^ ^]^ Aerobic glycolysis has been confirmed in GBM, and the resultant lactate accumulation is thought to contribute to GBM invasiveness, chemotherapy resistance, and GSC maintenance.^[^ ^18^, ^19^, ^20^ ^]^ Recent studies have demonstrated that lactate can also act as a substrate for the post‐translational modification of protein lysine residues, known as lysine lactylation (Kla), which directly regulates protein function.^[^ ^21^ ^]^ Histone lactylation at H3K18 (H3K18la) directly promotes gene transcription and participates in macrophage M1/2 polarization, somatic cell reprogramming, and tumorigenesis.^[^ ^21^, ^22^ ^]^ For example, lactate accumulated in the tumor microenvironment promotes methyltransferase 3 (METTL3) expression in tumor‐infiltrating myeloid cells via H3K18la, inducing an immunosuppressive effect through the METTL3/m^6^A/JAK1/STAT3 pathway.^[^ ^23^ ^]^ H3K18la also promotes tumorigenesis by enhancing the transcriptional expression of human YTH N6‐methyladenosine RNA‐binding protein F2 (YTHDF2) in ocular melanoma.^[^ ^24^ ^]^ Thus, lactate‐derived histone lactylation links glucose metabolism with gene expression, highlighting its role in tumor biology.

To further elucidate the regulatory effects of lactate on GSCs, we screened for key molecules involved in lactate‐mediated regulation of GSC stemness using public and internal databases and identified vaccinia‐related kinase 1 (VRK1) as a key molecule. VRK1, a nuclear serine/threonine kinase, binds to various chromosomal proteins, including histones, transcription factors, and DNA damage repair proteins, to form stable complexes.^[^ ^25^ ^]^ As a chromatin kinase, VRK1 modulates the expression of multiple signaling molecules and transcription factors, such as tumor protein p53 (TP53),^[^ ^26^ ^]^ activating transcription factor 2 (ATF2),^[^ ^27^ ^]^ and c‐Jun,^[^ ^28^ ^]^ which are implicated in tumor initiation and progression. Acting as a chromatin remodeling enzyme, VRK1 phosphorylates histones, thereby influencing their acetylation and methylation status to regulate gene transcription, DNA damage response, and the cell cycle.^[^ ^29^, ^30^ ^]^ VRK1 is overexpressed in various tumor types and is associated with an unfavorable prognosis.^[^ ^31^, ^32^, ^33^, ^34^ ^]^ Its role in tumors is closely linked to its functions in cell proliferation, cell cycle regulation, and DNA damage repair signaling pathways.^[^ ^25^ ^]^ In glioma, existing research on VRK1 primarily focuses on its role in cell proliferation^[^ ^34^ ^]^ and DNA damage repair,^[^ ^35^ ^]^ while its regulatory mechanisms in glioma stemness remain largely unexplored.

This study aimed to explore the regulatory effects of lactate and histone lactylation on the stemness and proliferation of GSCs. We focused on VRK1 as a key molecule mediating lactate‐driven regulation of GSCs in GBM. We found that lactate promoted H3K18 lactylation at the *VRK1* promoter in GSCs, thereby upregulating VRK1 expression. Further research elucidated the specific mechanisms by which the VRK1/YBX1/SOX2 pathway regulates GSC stemness and proliferation. Additionally, we engineered a VRK1‐target nanoliposome (A/TMZ‐siVRK1) that effectively suppressed GSC stemness and proliferation, underscoring its therapeutic potential in GBM.

## 2 Results

### 2.1 Lactate Promotes the Stemness and Proliferation of GSCs in GBM

Given the critical role of lactate in tumor initiation and progression,^[^ ^36^ ^]^ we investigated its regulatory effects on GSC stemness and proliferation in GBM. In this study, we utilized four GSC cell lines (GSC4, GSC21, GSC40, and GSC63), which were derived from clinical GBM tissue specimens.^[^ ^37^, ^38^ ^]^ First, we examined the impact of lactate on stemness marker expression in GSCs. Following incubation of GSCs with 10 mm sodium lactate for 24 h, we observed a general upregulation of both mRNA and protein levels of stemness markers, including SOX2, SOX9, OLIG2, CD133, NES, and POU3F2 (Figure S1A–E, Supporting Information). Next, we assessed the effect of lactate on the stemness and proliferation capability of GSCs from a functional perspective. Neurosphere proliferation assay revealed that lactate increased the size of neurospheres formed by GSCs (Figure S1F, Supporting Information). Extreme limiting dilution analysis (ELDA) demonstrated that lactate enhanced the self‐renewal capability of GSCs (Figure S1G–I, Supporting Information). Neurosphere formation assay showed that lactate increased the number of neurospheres formed by GSCs (Figure S1J, Supporting Information). Together, these findings indicate that lactate upregulates stemness markers and promotes the proliferation and self‐renewal of GSCs.

Lactate is a crucial component of the tumor microenvironment. Monocarboxylate transporters 1/2 (MCT1/2) transport exogenous lactate from the tumor microenvironment into cells to modulate cellular function, while lactate dehydrogenase A (LDHA) enables endogenous lactate production by tumor cells.^[^ ^22^, ^39^ ^]^ To elucidate the source of lactate regulating GSC stemness and proliferation, we used the MCT1/2 inhibitor AR‐C155858 and the LDHA inhibitor (R)‐GNE‐140. Western blot analysis revealed that exogenous lactate increased SOX2 expression in GSCs, and this upregulation was significantly inhibited by AR‐C155858 (Figure S2A, Supporting Information). Functional assays showed that exogenous lactate enhanced proliferation, self‐renewal, and neurosphere formation of GSCs, whereas these promoting effects were significantly attenuated by AR‐C155858 (Figure S2B–E, Supporting Information). We next investigated whether endogenous lactate produced by LDHA contributes to the regulation of GSC stemness and proliferation. GSCs were incubated with PBS or 1 µm LDHA inhibitor (R)‐GNE‐140 for 24 h. Western blot analysis showed that (R)‐GNE‐140 significantly reduced SOX2 expression in GSCs (Figure S2F, Supporting Information). Additionally, (R)‐GNE‐140 inhibited proliferation, self‐renewal, and neurosphere formation of GSCs (Figure S2G–J, Supporting Information). Collectively, these findings demonstrate that both exogenous and endogenous lactate promote the stemness and proliferation of GSCs.

### 2.2 Lactate Regulates the Stemness and Proliferation of GSCs via VRK1

To identify the key molecules involved in lactate‐mediated regulation of GSC stemness, we conducted bioinformatics‐based gene screening (**Figure** **1**A). We analyzed differentially expressed genes between GBM and low‐grade glioma (LGG) using The Cancer Genome Atlas (TCGA) and Chinese Glioma Genome Atlas (CGGA) datasets, selecting genes with high expression levels in GBM (Log FC > 0.5, *p* < 10^−6^) (Figure S3A,B, Supporting Information). We also analyzed sequencing data from lactate‐treated GBM cell lines in the GSE145699 dataset,^[^ ^40^ ^]^ identifying 924 upregulated genes following lactate treatment (*p* < 0.01) (Figure S3C, Supporting Information). Additionally, we analyzed paired sequencing data from GSCs and DGCs in our internal dataset and screened for genes highly expressed in GSCs compared to DGCs (Log FC > 6, *p* < 10^−6^) (Figure S3D, Supporting Information). By integrating these datasets with the glioma‐intrinsic gene set^[^ ^41^ ^]^ and the gene set associated with proliferating stem‐like glioma cells,^[^ ^42^ ^]^ we identified overlapping candidate genes, including centrosomal protein 55 (*CEP55*), aurora kinase B (*AURKB*), NIMA‐related kinase 2 (*NEK2*), VRK1, cell division cycle associated gene 8 (*CDCA8*), kinesin family member C1 (*KIFC1*), and kinesin family member 14 (*KIF14*) (Figure S3E, Supporting Information). We treated GSCs with sodium lactate and assessed the mRNA levels of seven candidate genes using RT‐qPCR. Following lactate treatment, the mRNA levels of *CEP55*, *AURKB*, *NEK2*, *VRK1*, *CDCA8*, *KIFC1*, and *KIF14* were generally upregulated in GSCs, with *VRK1* showing the most significant increase (Figure S3F–I, Supporting Information). RNA sequencing data from the GSE145699 dataset showed high VRK1 expression in lactate‐treated GBM cell lines.^[^ ^40^ ^]^ Previous studies have reported that VRK1 regulates cell proliferation, cell cycle, and DNA damage repair‐related therapeutic resistance.^[^ ^25^ ^]^ Based on these results, we speculate that *VRK1* is a key gene in promoting the stemness and proliferation of GSCs through lactate regulation in GBM.

**Figure 1:** VRK1 regulates the stemness and proliferation of GSCs in vitro. A) Screening flowchart (authorized by BioRender) for identifying key genes involved in lactate‐mediated regulation of GSC stemness and proliferation in GBM. B) Stable transfected cell lines with *VRK1* knockdown were constructed using lentiviral shVRK1‐1 and shVRK1‐2 sequences in GSC4 and GSC63 cells, and the knockdown efficiency was verified by western blot. C) Neurosphere proliferation assay showed that *VRK1* knockdown reduced the size of neurospheres formed by GSCs (*n* = 3, Student's t‐test). D,E) ELDA showed that *VRK1* knockdown inhibited the self‐renewal capability of GSCs (*n* = 3). F) Neurosphere formation assay showed that *VRK1* knockdown decreased the number of neurospheres formed by GSCs (*n* = 3, Student's t‐test). G) Western blot verified the overexpression efficiency of VRK1 in GSC21 and GSC40 cells. H) Neurosphere proliferation assay showed that *VRK1* overexpression increased neurosphere size (*n* = 3, Student's t‐test). I,J) ELDA showed that *VRK1* overexpression enhanced the self‐renewal capacity of GSCs. K) Neurosphere formation assay showed that *VRK1* overexpression increased the number of neurospheres formed by GSCs (*n* = 3, Student's t‐test). Data were presented as mean ± SD, ^*^ *p* < 0.05, ^**^ *p* < 0.01, ^***^ *p* < 0.001, ^****^ *p* < 0.0001.

In our internal dataset, VRK1 was significantly overexpressed in GSCs compared to paired DGCs, with expression patterns consistent with those of SOX2 (Figure S4A, Supporting Information). VRK1 expression was relatively higher in GSC4 and GSC63 cells, and lower in GSC21 and GSC40 cells. We established stably transfected cell lines with *VRK1* knockdown in GSC4 and GSC63 cells and *VRK1* overexpression in GSC21 and GSC40 cells. The efficiency of *VRK1* knockdown and overexpression was verified by western blot (Figure 1B,G) and qPCR (Figure S4B,C, Supporting Information). *VRK1* knockdown reduced neurosphere size (Figure 1C), self‐renewal (Figure 1D,E), and neurosphere formation (Figure 1F). *VRK1* overexpression increased neurosphere size (Figure 1H), self‐renewal (Figure 1I,J), and neurosphere formation (Figure 1K). These results indicate that VRK1 promotes the proliferation and self‐renewal of GSCs in vitro.

In vivo, we established an orthotopic xenograft tumor model in nude mice using GSC63 cells with *VRK1* knockdown. Hematoxylin and eosin (H&E) staining revealed that *VRK1* knockdown inhibited intracranial tumor growth compared to the control group (**Figure** **2**A,B). Survival analysis demonstrated that *VRK1* knockdown significantly prolonged the survival time of nude mice (Figure 2C). Immunohistochemistry (IHC) revealed that *VRK1* knockdown inhibited the expression of the proliferation marker Ki67 (Figure 2D). In vivo limiting dilution assays further indicated that *VRK1* knockdown significantly impaired the intracranial tumorigenic potential of GSC63 cells (Figure 2E).

**Figure 2:** VRK1 regulates the stemness and proliferation of GSCs in vivo. A,B) An orthotopic xenograft tumor model was established in nude mice using GSC63 cells with *VRK1* knockdown. Fluorescence imaging (A) and H&E staining (B) showed that *VRK1* knockdown reduced intracranial tumor volume (*n* = 5). C) Kaplan‐Meier survival analysis indicated that *VRK1* knockdown prolonged survival (*n* = 5, Log‐Rank test). D) IHC staining of VRK1 and Ki67 in tumor tissues. E) In vivo limiting dilution assays revealed decreased tumorigenic potential of GSC63 cells following *VRK1* knockdown (*n* = 5). ^*^ *p* < 0.05, ^**^ *p* < 0.01.

We next analyzed the correlation between *VRK1* and common stemness markers *SOX2*, *SOX9*, *OLIG2*, *NES*, and *POU3F2* in the CGGA dataset. Among these, *SOX2* exhibited the strongest correlation with *VRK1* (**Figure** **3**A). *VRK1* knockdown downregulated both mRNA and protein expression of SOX2 in GSC4 and GSC63 cells (Figure 3B,C), while *VRK1* overexpression upregulated both mRNA and protein expression of SOX2 in GSC21 and GSC40 cells (Figure S4D,E, Supporting Information). These findings suggest that VRK1 regulates SOX2 expression at the transcriptional level, thereby influencing the stemness and proliferation of GSCs.

**Figure 3:** Lactate regulates the stemness and proliferation of GSCs via *VRK1*. A) Correlation analysis of *VRK1* with stemness markers in the CGGA dataset: *NES* (r = 0.1200), *OLIG2* (r = 0.2529), *POU3F2* (r = 0.3106), *PROM1* (r = 0.1061), *SOX2* (r = 0.4248), and *SOX9* (r = 0.3319) (*n* = 137, Pearson correlation). B) RT‐qPCR analysis revealed that *VRK1* knockdown significantly decreased the mRNA level of SOX2 (*n* = 3, Student's t‐test). C) Western blot showed that *VRK1* knockdown reduced the protein level of SOX2. D) Western blot revealed that lactate failed to upregulate SOX2 expression in GSCs following *VRK1* knockdown. E,F) ELDA showed that lactate failed to enhance the self‐renewal capacity in GSCs following *VRK1* knockdown (*n* = 3). G) Neurosphere proliferation assay indicated that lactate failed to increase neurosphere size in GSCs following *VRK1* knockdown (*n* = 3, One‐way ANOVA test). H) Neurosphere formation assay indicated that lactate failed to promote neurosphere formation in GSCs following *VRK1* knockdown (*n* = 3, One‐way ANOVA test). Data were presented as mean ± SD, ns *p* > 0.05, ^*^ *p* < 0.05, ^**^ *p* < 0.01, ^***^ *p* < 0.001, ^****^ *p* < 0.0001.

To confirm whether lactate‐mediated stemness and proliferation regulation of GSCs depend on VRK1, we treated GSC4 and GSC63 cells with sodium lactate following *VRK1* knockdown. The lactate‐induced increase in SOX2 expression was inhibited by *VRK1* knockdown in GSCs (Figure 3D), indicating that lactate regulates SOX2 expression via *VRK1*. Additionally, lactate failed to enhance self‐renewal capability (Figure 3E,F), neurosphere size (Figure 3G), and neurosphere formation (Figure 3H) in GSCs after *VRK1* knockdown. These results reveal that lactate regulates the stemness and proliferation of GSCs via *VRK1*.

### 2.3 Lactate Regulates VRK1 Expression Through H3K18la in GSCs

Histone lactylation, derived from lactate, is a novel protein modification process that regulates the proliferation and invasion of tumor cells, as well as modulates immune cells to form an immunosuppressive microenvironment. We further investigated whether lactate mediates its effects on GSCs via histone lactylation. Western blot revealed that lactate increased overall Kla levels in GSCs, concomitantly upregulating VRK1 and SOX2 expression (**Figure** **4**A). Lactate elevated both mRNA and protein levels of VRK1. To assess whether VRK1 itself undergoes lactylation, we performed co‐immunoprecipitation (Co‐IP) experiments in GSC4 and GSC63 cells using VRK1 and pan anti‐Kla antibody. The results revealed that VRK1 itself did not undergo lactylation (Figure S5A, Supporting Information). After treatment with various lactate concentrations (0, 5, 10, and 20 mm) for 24 h, pan‐lysine lactylation and common histone lactylation modifications were elevated in GSCs, with the highest degree of lactylation observed at 10 mm lactate (Figure S5B, Supporting Information). Additionally, GSCs were treated with 10 mm lactate, and lactylation levels were assessed at different time points (0, 12, 24, and 48 h), with the highest degree of lactylation observed at 24 h (Figure S5C, Supporting Information). Given that histone epigenetic modification plays a crucial role in transcriptional regulation, we hypothesized that lactate might regulate VRK1 expression through histone lactylation. To identify which histone lactylation modification is dominant, we performed IP and found that H3 histone lactylation was most significantly enhanced in GSC4 cells following lactate treatment (Figure 4B). Western blotting with antibodies targeting H3K9la, H3K14la, H3K18la, and H3K56la demonstrated that H3K18la exhibited the most pronounced upregulation in response to lactate in GSCs (Figure 4C). These results indicate that lactate promotes histone lactylation in GSCs, particularly at the H3K18 site, suggesting that lactate may regulate the stemness and proliferation of GSCs through H3K18la. We further performed CUT&Tag to detect DNA fragments bound to the H3K18la antibody. CUT&Tag revealed that H3K18la bound to the *VRK1* promoter region, but not to the *SOX2* gene fragment (Figure 4D). Chromatin immunoprecipitation (ChIP) further confirmed that H3K18la bound to the *VRK1* promoter region in GSC4 and GSC63 cells (Figure 4E,F), indicating that lactylation modification occurrs at the 18^th^ lysine residue of H3 histone within the *VRK1* promoter region.

**Figure 4:** Lactate regulates VRK1 expression by inducing H3K18la in GSCs. A) Western blot revealed increased levels of overall Kla, VRK1, and SOX2 in GSCs treated with lactate (sodium lactate, 10 mm, 24 h). B) IP indicated that H3 histone lactylation was the most significant enhancement compared with other histones following lactate treatment in GSC4 cells. C) Western blot showed the expression levels of H3K9la, H3K14la, H3K18la, and H3K56la in GSCs treated with lactate or PBS. D) CUT&Tag indicated that the H3K18la antibody bound to the *VRK1* promoter in GSC63 cells. E,F) ChIP confirmed that H3K18la antibody bound to the *VRK1* promoter in GSC4 and GSC63 cells (*n* = 3, Student's t‐test). G) Western blot showed that C646 (100 µm, 24 h) significantly reduced H3K18la levels and downregulated VRK1 and SOX2 expression, whereas TSA (1 µm, 24 h) increased H3K18la levels and upregulated VRK1 and SOX2 expression. H) MCT1/2 inhibitor AR‐C155858 inhibited the upregulation of H3K18la, VRK1, and SOX2 induced by exogenous lactate in GSCs (AR‐C155858, 1 mm, 24 h). I) LDHA inhibitor (R)‐GNE‐140 reduced H3K18la levels and downregulated VRK1 and SOX2 in GSCs ((R)‐GNE‐140, 1 µm, 24 h). Data were presented as mean ± SD, ^**^ *p* < 0.01, ^****^ *p* < 0.0001.

Acetyltransferase p300, a lactylation‐modifying enzyme, increases lactylation levels, whereas histone deacetylase (HDAC), a delactylation‐modifying enzyme, reduces lactylation levels.^[^ ^23^, ^43^ ^]^ To further explore the regulation of VRK1 expression by histone lactylation, we used the p300 inhibitor C646 to decrease lactylation levels and the HDAC inhibitor trichostatin A (TSA) to enhance lactylation. GSCs were treated with or without 10 mm sodium lactate, 100 µm p300 inhibitor C646, or 1 µm HDAC inhibitor TSA for 24 h. C646 significantly reduced H3K18la levels and downregulated VRK1 and SOX2 expression, whereas TSA increased H3K18la levels and upregulated VRK1 and SOX2 expression (Figure 4G). These results indicate that lactate accumulated in the tumor microenvironment is sufficient to induce VRK1 and SOX2 expression through H3K18la.

To verify the regulatory effects of exogenous and endogenous lactate on histone lactylation, we used the MCT1/2 inhibitor AR‐C155858 and the LDHA inhibitor (R)‐GNE‐140. Exogenous lactate increased H3K18la lactylation levels in GSCs, and the upregulation of H3K18la, VRK1, and SOX2 induced by exogenous lactate was significantly inhibited by AR‐C155858 (Figure 4H). Additionally, (R)‐GNE‐140 reduced H3K18la levels and downregulated VRK1 and SOX2 expression in GSCs (Figure 4I). Both endogenous and exogenous lactate promote histone lactylation, thereby regulating the expression of VRK1 and SOX2.

### 2.4 VRK1 Enhances YBX1 Protein Stability and Promotes Its Phosphorylation

We overexpressed *VRK1* in GSC40 cells using lentiviral transfection and performed Co‐IP with an anti‐VRK1 antibody. Mass spectrometry analysis of the Co‐IP products identified 184 proteins that specifically bind to VRK1 (Table S1, Supporting Information). Notably, SOX2 was not among these proteins, and Co‐IP further confirmed that VRK1 and SOX2 did not directly interact in GSC4 and GSC63 cells (Figure S6A, Supporting Information). Given that VRK1 regulates SOX2 expression at the transcriptional level, we hypothesized that VRK1 might modulate SOX2 expression through a transcription factor. By intersecting the 184 VRK1‐binding proteins with the glioma‐intrinsic gene set^[^ ^41^ ^]^ and the transcription factor gene set,^[^ ^44^ ^]^ we identified 12 transcription factors that bind to VRK1 (**Figure** **5**A). Correlation analysis between *SOX2* and these 12 transcription factors in GSCs using sequencing data from our internal glioma database and the GSE67089 database revealed that only Y‐box binding protein 1 (*YBX1*) met the criteria of Pearson r > 0.8 and *p* < 0.05 in both databases, indicating a strong positive correlation between *YBX1* and *SOX2* in GSCs (Figure 5B; Figure S6B, Supporting Information). In contrast, this correlation was not observed in DGCs (Figure S6C,D, Supporting Information), suggesting that the regulation of SOX2 by YBX1 is unique to GSCs. Co‐IP confirmed that VRK1 directly bound to YBX1 in GSC4 and GSC63 cells (Figure 5C). These results suggest that VRK1 regulates SOX2 expression via YBX1 in GSCs.

**Figure 5:** VRK1 directly binds to YBX1 and increases its protein stability. A) A Venn diagram showed the overlapping genes among the VRK1‐specific binding molecules, the glioma intrinsic expression gene set, and the transcription factor gene set. B) Correlation analysis between *SOX2* and 12 transcription factors in GSCs using sequencing data from the internal glioma database. C) Co‐IP revealed direct binding between VRK1 and YBX1 in GSC4 and GSC63 cells. D,E) RT‐qPCR analysis revealed that the mRNA level of YBX1 was not significantly altered following *VRK1* knockdown or overexpression in GSCs (*n* = 3, Student's t‐test). F) Western blot revealed that *VRK1* knockdown decreased YBX1 protein expression, and *VRK1* overexpression increased YBX1 protein expression. G) The protein degradation of YBX1 significantly slowed down over time after adding CHX in GSCs with *VRK1* overexpression compared to the controls. H) Western blot showed that MG132 (10 µm, 6 h) reduced YBX1 degradation in GSCs with *VRK1* knockdown, while 3‐MA (10 µm, 6 h) had no effect. I) Western blot demonstrated that YBX1 expression was significantly upregulated in GSCs with normal VRK1 expression following MG132 treatment, which was consistent with YBX1 expression in VRK1‐overexpressing GSCs treated with DMSO. J) IP demonstrated that the ubiquitination level of YBX1 significantly increased after *VRK1* knockdown and decreased after *VRK1* overexpression in GSCs treated with MG132. K) GST pull‐down assay validated the direct binding between VRK1 and YBX1. L) GST pull‐down assay revealed that YBX1 bound to wild‐type VRK1 but not to the K71‐mutant VRK1. Data were presented as mean ± SD, ns *p* > 0.05.

Knockdown or overexpression of *VRK1* altered YBX1 protein levels, but did not significantly affect its mRNA levels (Figure 5D–F), indicating that VRK1 may regulate the protein stability of YBX1. We treated VRK1‐overexpressing GSCs with 50 µg/mL of the protein synthesis inhibitor cycloheximide (CHX) for 0, 3, and 6 h. In the control group, YBX1 protein levels decreased over time following the addition of CHX. However, in VRK1‐overexpressing GSCs, YBX1 protein degradation was significantly weakened, indicating that VRK1 enhances the protein stability of YBX1 (Figure 5G). To determine which protein degradation pathway of YBX1 is affected by VRK1, we treated *VRK1*‐knockdown GSCs with the proteasome degradation inhibitor MG132 and the lysosome degradation inhibitor 3‐Methyladenine (3‐MA). YBX1 degradation was suppressed in *VRK1*‐knockdown GSCs treated with MG132, but not with 3‐MA, indicating that VRK1 reduces YBX1 degradation via the proteasome pathway (Figure 5H). YBX1 expression was significantly upregulated in GSCs with normal VRK1 expression following MG132 treatment, which was consistent with YBX1 expression in VRK1‐overexpressing GSCs treated with dimethyl sulfoxide (DMSO) (Figure 5I). These results suggest that VRK1 enhances YBX1 protein stability primarily through the proteasome pathway. We further explored whether VRK1 binding to YBX1 inhibits its ubiquitination. GSC4 cells with *VRK1* knockdown and GSC21 cells with *VRK1* overexpression were treated with MG132, followed by IP, and YBX1 ubiquitination was detected using an anti‐ubiquitin (anti‐Ub) antibody. *VRK1* knockdown increased YBX1 ubiquitination without altering total YBX1 protein levels, whereas *VRK1* overexpression decreased YBX1 ubiquitination (Figure 5J). To further explore the ubiquitination sites of YBX1, we constructed HA‐tagged plasmids encoding wild‐type ubiquitin, K48 (ubiquitin mutant containing only K48 lysine), K48R, K63 (ubiquitin mutant containing only K63 lysine), and K63R, and transfected them into HEK293T cells. Under *VRK1* overexpression, YBX1 ubiquitination was reduced when tagged with wild‐type or K48 ubiquitin compared to wild‐type ubiquitin without *VRK1* overexpression, indicating that *VRK1* overexpression suppresses YBX1 ubiquitination. Additionally, HA‐labeled YBX1 ubiquitination was detected with wild‐type or K48 ubiquitin, but not with K63 ubiquitin, indicating that VRK1 specifically decreases K48‐linked YBX1 ubiquitination, but not K63‐linked ubiquitination (Figure S7A,Supporting Information). Consistently, YBX1 was resistant to K48R‐mediated ubiquitination under *VRK1* overexpression, further confirming that VRK1 regulates YBX1 ubiquitination at K48 (Figure S7A,Supporting Information). Together, these findings demonstrate that VRK1 reduces K48‐linked ubiquitination of YBX1, thereby stabilizing YBX1 and promoting GSC proliferation and stemness maintenance.

To confirm the direct binding of VRK1 to YBX1, we performed a glutathione S‐transferase (GST) pull‐down assay using purified GST‐VRK1 protein and recombinant YBX1 protein. YBX1 expression was detected in the GST‐VRK1 group but not in the GST‐only group, confirming that VRK1 directly binds to YBX1 (Figure 5K). Given that VRK1 is a serine/threonine kinase^[^ ^25^, ^45^ ^]^ and YBX1 can be phosphorylated at serine residues,^[^ ^46^ ^]^ we hypothesized that YBX1 binds to the active site of the VRK1 phosphatase. Lys71 is the catalytic residue within the VRK1 active site, and the K71M mutation eliminates VRK1 kinase activity.^[^ ^45^ ^]^ Therefore, we constructed a purified GST‐VRK1 K71M mutant protein and performed a GST pull‐down assay. In the wild‐type GST‐VRK1 group, YBX1 expression was detected, while in the GST‐VRK1 K71M group, YBX1 expression was not detected (Figure 5L). These results indicate that the kinase domain of VRK1 is crucial for maintaining the interaction between VRK1 and YBX1.

Previous studies have shown that phosphorylation of YBX1 at Ser102 is crucial for its nuclear translocation in cancer cells.^[^ ^47^, ^48^, ^49^ ^]^ We further investigated whether VRK1 can phosphorylate YBX1. In vitro kinase assay demonstrated that VRK1 phosphorylated YBX1 in a dose‐dependent manner. Specifically, the degree of YBX1 phosphorylation increased progressively with increasing concentrations of VRK1, under fixed concentrations of YBX1 and ATP (**Figure** **6**A,B). No YBX1 phosphorylation was detected in the VRK1 K71M mutant group (Figure 6B). *VRK1* knockdown decreased the levels of total YBX1 protein and phosphorylated YBX1 (Ser102), whereas *VRK1* overexpression increased the levels of total YBX1 protein and phosphorylated YBX1 (Ser102) (Figure 6C). Immunofluorescence further showed that *VRK1* knockdown reduced YBX1 expression in the nucleus, suggesting that *VRK1* knockdown suppresses YBX1 nuclear translocation in GSCs (Figure 6D). Nuclear‐cytoplasmic fractionation assays showed that *VRK1* knockdown reduced phosphorylated YBX1 (Ser102) and total YBX1 protein levels in both the cytoplasm and nucleus (Figure 6E). Compared with wild‐type VRK1 overexpression, GSCs overexpressing the VRK1 K71M mutant failed to exhibit elevated levels of phosphorylated YBX1 (Ser102) or total YBX1 protein in either the cytoplasm or nucleus (Figure 6F). To investigate the role of YBX1 Ser102 phosphorylation in nuclear translocation, we constructed a YBX1 S102 mutant (YBX1 S102A). Nuclear‐cytoplasmic fractionation assays revealed that GSCs overexpressing wild‐type YBX1 significantly increased the expression levels of YBX1 and phosphorylated YBX1 in the nucleus. In contrast, GSCs overexpressing YBX1 S102A did not show increased levels of YBX1 and phosphorylated YBX1 in the nucleus compared to the control group (Figure 6G). This indicates that phosphorylation of YBX1 at Ser102 is essential for its nuclear translocation in GSCs. Furthermore, GSCs overexpressing wild‐type YBX1 increased SOX2 expression, while GSCs overexpressing YBX1 S102A failed to do so (Figure 6H). Collectively, these results indicate that VRK1 phosphorylates YBX1 at Ser102 and promotes its nuclear translocation in GSCs.

**Figure 6:** VRK1 phosphorylates YBX1 to promote its nuclear translocation. A) In vitro kinase assay showed that VRK1 protein phosphorylated YBX1 in a dose‐dependent manner. B) In vitro kinase assay showed that the wild‐type VRK1 protein, but not the K71‐mutant VRK1 protein, phosphorylated YBX1 in a dose‐dependent manner. C) Western blot showed that *VRK1* knockdown decreased the protein levels of YBX1, phosphorylated YBX1 (Ser102), and SOX2, whereas *VRK1* overexpression increased their protein levels. D) Immunofluorescence revealed that *VRK1* knockdown reduced the nuclear expression of YBX1 in GSC4 and GSC63 cells. E) Western blot showed that *VRK1* knockdown or overexpression correspondingly decreased or increased YBX1, phosphorylated YBX1 (Ser102), and SOX2 protein levels in both the cytoplasm and nucleus of GSCs. F) YBX1 and phosphorylated YBX1 (Ser102) were increased in both the cytoplasm and nucleus of GSCs overexpressing wild‐type VRK1, whereas the K71‐mutant VRK1 showed no such effect. G) Nuclear‐cytoplasmic fractionation assays revealed that GSCs overexpressing wild‐type YBX1 increased YBX1 and phosphorylated YBX1 levels in the nucleus, whereas overexpressing YBX1 S102A did not increase YBX1 and phosphorylated YBX1 levels in the nucleus. H) GSCs overexpressing wild‐type YBX1 increased SOX2 expression, while GSCs overexpressing YBX1 S102A did not increase SOX2 expression.

### 2.5 VRK1/YBX1/SOX2 Pathway Regulates the Stemness of GSCs

We predicted the binding sequence of YBX1 to the *SOX2* promoter region using the JASPAR website and found that YBX1 could bind to the *SOX2* promoter at positions 362 to 354, thereby participating in the transcriptional regulation of *SOX2* (Figure S6E, Supporting Information). Based on this predicted site, we designed primers for ChIP, which confirmed that YBX1 bound to the *SOX2* promoter region (**Figure** **7**A). To further investigate whether VRK1 regulates the stemness and proliferation of GSCs via YBX1, we knocked down *YBX1* in VRK1‐overexpressing GSCs. The upregulation of SOX2 expression induced by VRK1 overexpression was attenuated by *YBX1* knockdown (Figure 7B). Neurosphere proliferation assay showed that *YBX1* knockdown inhibited the VRK1‐mediated increase in neurosphere size (Figure 7C). ELDA demonstrated that the promotion of self‐renewal in GSCs caused by VRK1 overexpression was effectively inhibited by *YBX1* knockdown (Figure 7D,E). Neurosphere formation assay showed that *YBX1* knockdown diminished the increase in neurosphere formation induced by VRK1 overexpression (Figure 7F). These results indicate that VRK1 regulates SOX2 expression and promotes the stemness and proliferation of GSCs via *YBX1*.

**Figure 7:** VRK1 regulates the stemness and proliferation of GSCs via *YBX1*. A) Ch‐IP revealed that YBX1 bound to the *SOX2* promoter region (*n* = 3, Student's t‐test). B) Western blot demonstrated that the upregulation of SOX2 expression caused by *VRK1* overexpression in GSCs was inhibited by *YBX1* knockdown. C) Neurosphere proliferation assay indicated that the promotion of neurosphere proliferation caused by *VRK1* overexpression in GSCs was inhibited by *YBX1* knockdown (*n* = 3, One‐way ANOVA test). D,E) ELDA showed that the promotion of self‐renewal caused by *VRK1* overexpression in GSCs was inhibited by *YBX1* knockdown (*n* = 3). F) Neurosphere formation assay demonstrated that the promotion of neurosphere formation induced by *VRK1* overexpression in GSCs was inhibited by *YBX1* knockdown (*n* = 3, One‐way ANOVA test). Data were presented as mean ± SD, ns *p* > 0.05, ^*^ *p* < 0.05, ^**^ *p* < 0.01, ^***^ *p* < 0.001, ^****^ *p* < 0.0001.

Hypoxia and acidic stress are core features of the tumor microenvironment in GBM, which can promote GSC maintenance.^[^ ^17^ ^]^ To further investigate the effects of hypoxia on GSCs, we treated GSCs with 200 µm cobalt chloride for 24 h to mimic hypoxic conditions. Both hypoxia and lactate promoted the activation of the VRK1/YBX1/SOX2 pathway in both GSCs and DGCs (Figure S8A,B, Supporting Information). Under hypoxic conditions, GSCs exhibited enhanced stemness and proliferation compared to controls (Figure S8C–F, Supporting Information). Additionally, the expression levels of VRK1, YBX1, and SOX2 were upregulated in GSCs and DGCs under hypoxic conditions (Figure S8G,H Supporting Information). *VRK1* knockdown significantly inhibited the hypoxia‐induced enhancement of proliferation and self‐renewal in GSCs (Figure S8C–F, Supporting Information). Moreover, *VRK1* knockdown effectively attenuated the hypoxia‐induced upregulation of YBX1 and SOX2 in both GSCs and DGCs (Figure S8G,H, Supporting Information). These findings indicate that under both hypoxic and lactate conditions, VRK1 functions as a key regulator of the VRK1/YBX1/SOX2 pathway. The enhancement of stemness and proliferation in GSCs induced by hypoxia or lactate can be effectively reversed by *VRK1* knockdown.

We further examined the expression of VRK1, YBX1, and SOX2 in clinical glioma tissue specimens. Immunohistochemistry revealed that VRK1 and YBX1 were localized to both the nucleus and cytoplasm, whereas SOX2 was predominantly expressed in the nucleus (**Figure** **8**A). The expression levels of VRK1, YBX1, and SOX2 were significantly elevated in GBM tissues, with median immunoreactive scores (IRS) of 9, 12, and 9, respectively. In contrast, these proteins were only weakly expressed in non‐tumor tissues adjacent to extensively resected gliomas, with a median IRS of 1 for all three proteins. The expression levels of VRK1, YBX1, and SOX2 increased with the pathological grade of glioma. The median IRS values for VRK1, YBX1, and SOX2 in grade II glioma tissues were 2, 3, and 2, respectively, whereas in grade III glioma tissues, the median IRS values were 4, 7, and 4, respectively (Figure 8A,B). Correlation analysis demonstrated positive correlations among VRK1, YBX1, and SOX2 expression in both glioma and GBM tissues (Figure 8C,D). These findings confirm that VRK1, YBX1, and SOX2 are overexpressed in GBM and suggest a regulatory relationship among them, consistent with previous research findings.

**Figure 8:** VRK1, YBX1, and SOX2 are highly expressed and exhibit a positive correlation in GBM. A) IHC staining showed that VRK1 and YBX1 were localized in both the nucleus and cytoplasm, while SOX2 was predominantly localized in the nucleus (Scale bars: 200, 50 µm). VRK1, YBX1, and SOX2 were weakly expressed in non‐tumor tissues but were significantly overexpressed in GBM, with expression levels increasing with glioma grade. B) IRS values of VRK1, YBX1, and SOX2 (Non‐tumor tissue: *n* = 3, WHO II glioma: *n* = 14, WHO III glioma: *n* = 12, GBM: *n* = 15; one‐way ANOVA test). C) Correlation analysis indicated that the expression levels of VRK1, YBX1, and SOX2 were positively correlated in glioma tissues (VRK1 versus YBX1, r = 0.8289, *p* < 0.0001; VRK1 versus SOX2, r = 0.8616, *p* < 0.0001; YBX1 versus SOX2, r = 0.8807, *p* < 0.0001; Pearson correlation). D) The expression levels of VRK1, YBX1, and SOX2 were positively correlated in GBM tissues (VRK1 versus YBX1, r = 0.5174, *p* = 0.0482; VRK1 versus SOX2, r = 0.6939, *p* = 0.0041; YBX1 versus SOX2, r = 0.5510, *p* = 0.0332; Pearson correlation). Data were presented as mean ± SD, ns *p* > 0.05, ^*^ *p* < 0.05, ^**^ *p* < 0.01, ^***^ *p* < 0.001, ^****^ *p* < 0.0001.

### 2.6 Preparation and Characterization of A/TMZ‐siVRK1

In this study, we designed a siVRK1‐based nanoliposome, A/TMZ‐siVRK1, to target VRK1 and enhance its synergistic effect with TMZ. A/TMZ‐siVRK1 was prepared via nanoprecipitation by incorporating TMZ and DOTAP‐siVRK1 into the hydrophobic core, while PEG_2000_‐DSPE, cholesterol, and angiopep‐2‐PEG_2000_‐DSPE constituted the lipid shell. For controls, we prepared phospholipid‐coated TMZ (A/TMZ‐siNC) and phospholipid‐coated poly (lactic‐co‐glycolic acid, PLGA) (A/PLGA‐siVRK1). Dynamic light scattering analysis showed that the particle diameters of TMZ‐siVRK1, A/TMZ‐siNC, A/PLGA‐siVRK1, and A/TMZ‐siVRK1 were 107.9±1.78 nm, 127.57±1.90 nm, 131.6±1.47 nm, and 133.27±1.00 nm, respectively (**Figure** **9**A). Transmission electron microscopy (TEM) imaging of TMZ‐siVRK1, A/TMZ‐siNC, A/PLGA‐siVRK1, and A/TMZ‐siVRK1 revealed clear core‐shell structures, with lipid molecules located on the outer layer of A/TMZ‐siVRK1 (Figure 9B). The zeta potentials of TMZ‐siVRK1, A/TMZ‐siNC, A/PLGA‐siVRK1, and A/TMZ‐siVRK1 were +12±1.14 mV, +8.27±1.42 mV, +7.83±1.3 mV, and +8.63±1.59 mV, respectively (Figure 9C). Agarose gel electrophoresis demonstrated that siVRK1 was completely adsorbed by DOTAP at an N/P ratio of 10:1 (Figure 9D), which was used for subsequent experiments. The serum stability of TMZ‐siVRK1, A/TMZ‐siNC, A/PLGA‐siVRK1, and A/TMZ‐siVRK1 was assessed in DMEM containing 10% fetal bovine serum (FBS), and no significant changes in size were observed over 6 days, indicating good serum stability of these nanoliposomes in 10% FBS (Figure 9E). Considering the weak acidity of the tumor microenvironment in vivo,^[^ ^50^ ^]^ changes in drug release from A/TMZ‐siVRK1 were tested using PBS at pH 6.5. The cumulative release profiles of TMZ and siVRK1 showed that the drug release from A/TMZ‐siVRK1 at pH 6.5 was higher than at pH 7.4 (Figure 9F,G). At pH 6.5, TMZ hydrolysis reached 71.12%±2.73% and siVRK1 hydrolysis reached 70.98%±3.99% within 24 h (Figure 9F,G). In contrast, at pH 7.4, TMZ hydrolysis reached 24.50%±3.08% and siVRK1 hydrolysis reached 25.13%±3.15% within 24 h (Figure 9F,G), revealing that the weakly acidic tumor microenvironment enhances drug release from nanoliposomes.

**Figure 9:** Synthesis and characterization of A/TMZ‐siVRK1. A) Size distribution of TMZ‐siVRK1, A/TMZ‐siNC, A/PLGA‐siVRK1, and A/TMZ‐siVRK1. B) TEM images of TMZ‐siVRK1, A/TMZ‐siNC, A/PLGA‐siVRK1, and A/TMZ‐siVRK1. C) Zeta potential of TMZ‐siVRK1, A/TMZ‐siNC, A/PLGA‐siVRK1, and A/TMZ‐siVRK1. D) Agarose gel electrophoresis experiments demonstrated that when the N/P ratio was 10:1, siVRK1 was completely adsorbed by DOTAP. E) Serum stability of TMZ‐siVRK1, A/TMZ‐siNC, A/PLGA‐siVRK1, and A/TMZ‐siVRK1 (*n* = 3). F,G) In vitro TMZ (F) or siVRK1 (G) drug release profiles under pH 6.5 or 7.4 PBS conditions (*n* = 3). H) The CLSM images were performed to test the ability of TMZ‐siVRK1‐FITC and A/TMZ‐siVRK1‐FITC to penetrate the BBB and target GSC63 (*n* = 3, Student's t‐test). Red: Dil‐labeled BBB layer cell membrane (HBMEC). Blue: DAPI‐labeled nuclei; green: TMZ‐siVRK1‐FITC or A/TMZ‐siVRK1‐FITC (FITC signal). Scale bar = 25 µm. I) CLSM images showing endosomal escape of A/TMZ‐siVRK1 in GSC63. Cells were incubated with A/TMZ‐siVRK1 at 37 °C for 1, 4, and 8 h. FITC‐labeled A/TMZ‐siVRK1 (green signal) was used. Nuclei were stained by DAPI (blue signal), and endosomes were stained with LysoTracker (red signal). Scale bars = 10 µm. J–L) The corresponding colocalization fluorescence intensity profiles of FITC (green) and endosomes (red) in GSC63 after FITC‐labeled A/TMZ‐siVRK1 treatment for 1 h (J), 4 h (K), and 8 h (L). M) The corresponding colocalization ratios of FITC (green) and endosomes (red) (*n* = 3, one‐way ANOVA test). N) Fluorescent image of TMZ‐siVRK1‐Cy5 and A/TMZ‐siVRK1‐Cy5 brain distribution in vivo was observed with a small animal imaging system at post‐injection 6, 12, and 24 h (left). Statistical analysis of fluorescence content of A/TMZ‐siVRK1‐Cy5 in mice brains with imaging in vivo (right) (*n* = 3, Student's t test). Data were presented as mean ± SD, ^*^ *p* < 0.05, ^**^ *p* < 0.01, ^***^ *p* < 0.001, ^****^ *p* < 0.0001.

To ensure therapeutic efficacy, selective uptake of nanoliposomes by glioma cells is essential. Angiopep‐2, a specific ligand for low‐density lipoprotein receptor‐related protein‐1 (LRP‐1), is highly expressed in both the blood‐brain barrier (BBB) and glioma cells. It has been widely used to modify nanoliposomes for targeted molecular therapy to increase drug concentration in GBM.^[^ ^50^ ^]^ Therefore, we modified the surface of TMZ‐siVRK1 using angiopep‐2 to enhance its distribution within glioma cells. As penetrating the BBB remains a critical challenge for drugs entering the central nervous system,^[^ ^50^ ^]^ effective transport of nanoliposomes across the BBB is essential for improving the therapeutic efficacy of gliomas. To evaluate the targeting capability of A/TMZ‐siVRK1, we established an in vitro BBB model to assess whether A/TMZ‐siVRK1‐FITC could traverse the endothelial barrier (Figure 9H). In the Transwell system, human brain microvascular endothelial cells (HBMECs) were cultured at the bottom of the upper chamber, and GSC63 cells were cultured at the bottom of the lower chamber. When the transendothelial electrical resistance (TEER) reached 200 Ω•cm^2^, the formation of the BBB was considered successful. The average fluorescence intensity of FITC in GSC63 cells treated with A/TMZ‐siVRK1‐FITC was significantly higher than that in cells treated with TMZ‐siVRK1‐FITC, with penetration rates of 68.32%±3.35% and 26.8%±5.38%, respectively (Figure 9H). These results demonstrate that angiopep‐2 modification effectively enhanced the BBB penetration capability of A/TMZ‐siVRK1‐FITC (Figure 9H).

Drugs are often sequestered in endosomal vesicles and degraded in the lysosomal lumen, leading to treatment failure. Therefore, we evaluated the endosomal escape capability of A/TMZ‐siVRK1‐FITC. After 8 h, the separation between the green and red fluorescence spots was more pronounced, and the colocalization ratio of labeled endosomes/lysosomes and A/TMZ‐siVRK1‐FITC was 38.57 ± 5.10%, indicating that A/TMZ‐siVRK1‐FITC could effectively escape from the endosomes, thereby ensuring the therapeutic efficacy of siVRK1 and TMZ (Figure 9I–M). To evaluate the targeting efficacy, we administered A/TMZ‐siVRK1‐Cy5 to mice bearing glioma cells (Figure 9N). Due to the targeting effect of angiopep‐2, A/TMZ‐siVRK1‐Cy5 exhibited significantly stronger Cy5 fluorescence intensity in gliomas compared to the TMZ‐siVRK1‐Cy5 group, which lacked angiopep‐2 modification (Figure 9N).

### 2.7 In Vivo Distribution, Pharmacokinetics, Biocompatibility, and Therapeutic Effect of A/TMZ‐siVRK1

To assess the in vivo metabolic profiles of TMZ‐siVRK1 and A/TMZ‐siVRK1, we utilized small animal imaging to track the distribution of TMZ‐siVRK1‐Cy5 and A/TMZ‐siVRK1‐Cy5 in the heart, liver, spleen, lungs, and kidneys. Both TMZ‐siVRK1‐Cy5 and A/TMZ‐siVRK1‐Cy5 exhibited significant accumulation in the liver, kidneys, and lungs, indicating clearance through these three organs (Figure S9A,B, Supporting Information). Following tail vein injection of TMZ and A/TMZ‐siVRK1, the pharmacokinetics of TMZ in an orthotopic xenograft tumor model were investigated using ultra‐performance liquid chromatography‐tandem mass spectrometry (UPLC‐MS/MS). The results revealed that after tail vein injection of free TMZ, its half‐life in plasma was 2.46 h. After injection of A/TMZ‐siVRK1, the half‐life of TMZ in plasma was extended to 8.41 h (Figure S9C, Supporting Information). Compared to TMZ‐siVRK1, there was a significant increase in TMZ content in GBM tissue after tail vein injection of A/TMZ‐siVRK1, while the TMZ content in normal brain tissue was reduced after tail vein injection of A/TMZ‐siVRK1 (Figure S9D,E, Supporting Information).

Furthermore, the pharmacokinetics of siVRK1 were assessed in an orthotopic xenograft tumor model using FITC‐labeled siVRK1 (siVRK1‐FITC). Following tail vein injection of free siVRK1, the plasma half‐life of siVRK1‐FITC was 2.07 h, and only a small amount of siVRK1‐FITC fluorescence was detected in the GBM tissue. Following tail vein injection of A/TMZ‐siVRK1, the half‐life of siVRK1‐FITC in plasma was prolonged to 5.70 h. Compared to TMZ‐siVRK1, stronger siVRK1‐FITC fluorescence was observed in GBM tissue after tail vein injection of A/TMZ‐siVRK1, while siVRK1‐FITC fluorescence in normal brain tissue was reduced (Figure S9F–H, Supporting Information).

To evaluate the potential toxic side effects of A/TMZ‐siVRK1, treatment was administered continuously for 8 days after establishing the patient‐derived xenograft model. On day 24, mice from each group were euthanized, and major organs were harvested for tissue paraffin sectioning and H&E staining. The results showed that the cardiac, hepatic, splenic, pulmonary, and renal tissue sections from the TMZ‐siVRK1, A/TMZ‐siNC, A/PLGA‐siVRK1, and A/TMZ‐siVRK1 groups exhibited no significant histological damage or morphological changes compared with the PBS group (Figure S10A, Supporting Information), indicating good biocompatibility and safety of A/TMZ‐siVRK1 in vivo. On the 7th day after treatment, blood was collected via tail vein puncture for routine hematological and biochemical analyses. The hematological markers and serum levels of alkaline phosphatase, alanine aminotransferase, aspartate aminotransferase, creatinine, and blood urea nitrogen in the TMZ‐siVRK1, A/TMZ‐siNC, A/PLGA‐siVRK1, and A/TMZ‐siVRK1 groups were not significantly different from those in the PBS group (*p* > 0.05) (Figure S10B, Supporting Information). Collectively, these results suggest that A/TMZ‐siVRK1 exhibits favorable biological safety in vivo.

### 2.8 Therapeutic Efficacy of A/TMZ‐siVRK1 in Glioma Models

To investigate the anti‐glioma activity of A/TMZ‐siVRK1, neurosphere formation and apoptosis assays were performed in GSC63 cells. The number of neurospheres decreased and the proportion of apoptotic cells increased in the A/TMZ‐siVRK1 group, indicating higher cytotoxicity of A/TMZ‐siVRK1 than that in the other groups (**Figure** **10**A,B). The in vivo therapeutic efficacy of combined siVRK1 and TMZ was evaluated using an intracranial tumor xenograft transplantation model constructed with GSC63 cells in BALB/c nude mice (Figure 10C). A/TMZ‐siVRK1 markedly suppressed intracranial tumor growth in BALB/c nude mice. The median survival time for GSC63‐bearing mice was 68 days for A/TMZ‐siVRK1, 45 days for A/PLGA‐siVRK1, 34 days for A/TMZ‐siNC, 32 days for TMZ‐siVRK1, and 31 days for PBS (Figure 10D). Mice treated with A/TMZ‐siVRK1 exhibited significantly extended survival time compared with all other treatments. Fluorescence imaging demonstrated that A/TMZ‐siVRK1 significantly inhibited intracranial tumor growth and reduced fluorescence intensity compared to the other groups (Figure 10E). These results were further confirmed by H&E staining (Figure 10F). Immunohistochemistry showed that the expression levels of VRK1, YBX1, and SOX2 were significantly reduced in the A/TMZ‐siVRK1 group compared to those in the PBS, TMZ‐siVRK1, A/TMZ‐siNC, and A/PLGA‐siVRK1 groups, indicating that A/TMZ‐siVRK1 inhibited VRK1/YBX1/SOX2 signal activation in gliomas (Figure 10G). The number of Ki‐67‐positive cells was the lowest in gliomas treated with A/TMZ‐siVRK1 (Figure 10G). These results demonstrate that the combination of TMZ with siVRK1 delivered by A/TMZ‐siVRK1 effectively inhibits glioma growth.

**Figure 10:** A/TMZ‐siVRK1 effectively inhibits glioma growth in vitro and in vivo. A) Neurosphere formation assay showed that the number of neurospheres formed by GSC63 cells treated with A/TMZ‐siVRK1 was decreased compared with PBS, TMZ‐siVRK1, A/TMZ‐siNC, and A/PLGA‐siVRK1 groups (*n* = 3, one‐way ANOVA test). B) Flow cytometry showed that the apoptosis rate of GSC63 cells treated with A/TMZ‐siVRK1 was increased compared with PBS, TMZ‐siVRK1, A/TMZ‐siNC, and A/PLGA‐siVRK1 groups (*n* = 3, one‐way ANOVA test). C) Experimental schedule of patient‐derived GSC63 inoculation and drug administration of PBS, TMZ‐siVRK1, A/TMZ‐siNC, A/PLGA‐siVRK1, and A/TMZ‐siVRK1. D) Kaplan–Meier survival curves of mice implanted with GSC63 cells (*n* = 5, Log‐rank test). E,F) In vivo fluorescence imaging (E) and H&E‐staining (F) of orthotopic xenograft tumor model. G) Immunohistochemical staining of VRK1, YBX1, SOX2, and Ki67 in glioma tissues of nude mice (Scale bar: 50 µm). Data were presented as mean ± SD, ^*^ *p* < 0.05, ^**^ *p* < 0.01, ^***^ *p* < 0.001, ^****^ *p* < 0.0001.

## 3 Discussion

Metabolic reprogramming is a hallmark of tumors, enabling tumor cells to rapidly proliferate by altering their energy metabolism to adapt to the hypoxic, acidic, and nutrient‐deficient tumor microenvironment. This process, characterized by enhanced glycolysis, abnormal mitochondrial metabolism, and lactate production, supplies essential metabolites for tumor cell proliferation.^[^ ^51^ ^]^ The Warburg effect, a hallmark of cancer metabolism, is one of the most extensively studied models of tumor metabolic reprogramming. Glycolysis‐dependent metabolism in tumor cells positions lactate as a key player in energy metabolism reprogramming, enabling rapid energy generation. Elevated lactate levels directly create an acidic tumor microenvironment, thereby promoting tumor progression and metastasis. Additionally, lactate within the tumor microenvironment can induce immunosuppression and facilitate immune evasion, thereby supporting tumor survival and growth.^[^ ^51^ ^]^ GBM is characterized by significant lactate accumulation.^[^ ^52^ ^]^ In human GBM cell lines U‐87 MG, A‐172, and U‐251 MG, lactate significantly enhanced cell proliferation, migration, and colony formation.^[^ ^53^ ^]^ GSCs have been identified as a subpopulation of tumor cells that drive treatment resistance and recurrence in GBM. However, studies on the role of lactate in regulating the stemness of GSCs remain limited. To further elucidate the regulatory effects of the glycolysis metabolite lactate on the stemness and proliferation of GSCs, as well as its key regulatory targets, we conducted this study. We discovered that in vitro lactate induction promoted the stemness and proliferation of GSCs, as well as upregulated the expression of stemness markers such as SOX2 and CD133. Lactate can also promote the expression of stemness markers in DGCs, thereby inducing a transition from a differentiated phenotype to a stem‐like state. These results expand the functional role of lactate in GSCs and further confirm that lactate is not merely a metabolic byproduct, but also a critical promoting factor in the development and progression of tumors. Further exploration of lactate functions and related pathways will provide deeper insights into the biological behavior of GBM.

To elucidate the specific mechanisms by which lactate regulates the stemness of GSCs in GBM, we performed bioinformatics analyses using clinical sequencing data from multiple public and internal databases. We identified VRK1 as a key regulator of lactate‐induced regulation of stemness and proliferation in GSCs. VRK1, a serine/threonine kinase, is overexpressed in various tumor types, including glioma, and is associated with poor prognosis.^[^ ^31^, ^32^, ^33^, ^34^ ^]^ Current research on VRK1 in glioma primarily focuses on cell proliferation^[^ ^34^ ^]^ and DNA damage repair,^[^ ^35^ ^]^ with limited exploration of its role in the stemness regulation of GSCs. Our study confirmed that VRK1 promotes the stemness and proliferation of GSCs both in vitro and in vivo, and regulates the expression of the stemness marker SOX2 at the transcriptional level. To determine whether lactate regulates stemness and proliferation via VRK1, we treated GSCs with lactate following *VRK1* knockdown and assessed their self‐renewal and proliferation capacity. These results confirm that lactate regulates the stemness and proliferation of GSCs via VRK1. Consistent with our findings, RNA sequencing data from the GSE145699 database showed increased VRK1 expression in GBM cells following lactate treatment.^[^ ^40^ ^]^ Clinical glioma tissue specimens revealed higher VRK1 expression in GBM compared to non‐tumor tissues and LGG, with expression levels increasing with pathological grade. Additionally, VRK1 expression in GBM was positively correlated with the expression of the stemness marker SOX2, supporting its role in stemness regulation. Given that GBM is characterized by significant lactate accumulation, we propose that high lactate levels contribute to VRK1 upregulation in GBM. Targeting VRK1 could be a potential therapeutic strategy to inhibit lactate‐driven stemness in GSCs.

Lactate‐derived histone lactylation is a novel epigenetic marker that has emerged as a research hotspot in oncology. Histone lactylation regulates various physiological processes, including transcriptional activation, cell reprogramming, pulmonary fibrosis, and macrophage polarization. Zhao et al. discovered that the mass shift of 72.021 Daltons at lysine residues in three proteolytic peptides was the same as that caused by the addition of a lactyl group to the ε‐amino group of lysine, providing the first evidence of histone Kla.^[^ ^21^ ^]^ Kla accumulates on specific gene promoters in cells stimulated by hypoxia, IFN‐γ, lipopolysaccharide, or cellular stress, directly regulating gene expression.^[^ ^21^, ^54^ ^]^ In tumor tissues, Kla promotes tumor immune evasion by inducing the anti‐inflammatory phenotype of tumor‐associated macrophages, and directly regulates oncogene expression to drive tumor growth, metastasis, and invasion.^[^ ^39^ ^]^ Our research demonstrated that lactate promotes histone lactylation in GSCs, with H3K18la showing the most significant response to lactate regulation. CUT&Tag and ChIP revealed that H3K18la binds to the *VRK1* promoter‐binding sequence in GSCs but not to the *SOX2* gene fragment. These findings indicate that lactate regulates VRK1 expression through histone lactylation at H3K18 in the *VRK1* promoter region, thereby modulating the stemness and proliferation of GSCs, which provides new evidence for the role of histone lactylation in regulating gene expression and tumorigenesis.

VRK1 interacts with various chromosomal proteins to form stable complexes, including histones, transcription factors, and DNA damage repair proteins.^[^ ^29^ ^]^ To elucidate the molecular mechanisms by which VRK1 regulates the stemness of GSCs, we performed Co‐IP combined with mass spectrometry to identify the molecules interacting with VRK1. Given that tumor stem cells often express high levels of stem cell‐related transcription factors to maintain their relevant characteristics, we further identified transcription factors significantly associated with SOX2 that specifically bind to VRK1 in GSCs. We found that VRK1 specifically bound to the transcription factor YBX1, which was further confirmed by Co‐IP. YBX1 is a transcription factor present in embryonic stem cells and various tumors.^[^ ^55^ ^]^ It is highly expressed in both GBM and neural stem cells.^[^ ^56^ ^]^ YBX1 has been reported to promote the growth of CSCs and regulate the expression of various stem cell‐related genes, including *SOX2*, *CD10*, *CD24*, and *CD44*.^[^ ^46^, ^57^ ^]^ Previous studies have shown that YBX1 can maintain the stemness of CSCs and reprogram differentiated cancer cells into CSCs.^[^ ^57^ ^]^ Our research confirms that YBX1 is highly expressed in GBM, and its expression positively correlates with the pathological grade of glioma, as well as with the expression of VRK1 and SOX2. We propose that VRK1 regulates SOX2 expression via YBX1. Notably, knockdown or overexpression of *VRK1* did not significantly alter the mRNA level of YBX1 but did affect its protein expression. Therefore, we explored the mechanisms by which VRK1 regulates YBX1 from two perspectives: protein stability and phosphorylation. We found that the interaction between VRK1 and YBX1 in GSCs reduces YBX1 ubiquitination and degradation, thereby increasing YBX1 protein stability and overall levels. Additionally, as a serine/threonine kinase, VRK1 can phosphorylate YBX1 at serine residues, promoting its nuclear translocation and transcriptional regulatory functions.^[^ ^58^, ^59^ ^]^ In vitro kinase assays demonstrated that VRK1 phosphorylated YBX1 in a dose‐dependent manner. *VRK1* knockdown inhibited YBX1 phosphorylation and nuclear translocation. These dual mechanisms regulate the stemness and proliferation of GSCs, providing a novel theoretical basis for the role of the VRK1/YBX1 axis in GSC regulation.

YBX1 is highly expressed in glioma tissues compared to adjacent normal brain tissues, with the highest expression levels observed in GBM.^[^ ^46^ ^]^ *YBX1* knockdown reduces the expression of the stemness marker SOX2, inhibits neurosphere growth, and suppresses tumor proliferation and invasion.^[^ ^56^ ^]^ Conversely, YBX1 expression is low in brain tumor‐initiating cells following induced differentiation.^[^ ^56^ ^]^ Given that both YBX1 and SOX2 are critical embryonic stem cell proteins, they appear to exhibit similar biological behavior.^[^ ^55^ ^]^ Studies have demonstrated a positive correlation between YBX1 and SOX2 expression in glioma cells.^[^ ^56^ ^]^ Our study confirmed that YBX1 and SOX2 were overexpressed in GBM and positively correlated. YBX1 bound to the *SOX2* promoter and regulated its transcriptional expression in GSCs. These findings are consistent with previous studies showing that YBX1 transcriptionally regulates SOX2 expression in esophageal squamous cell carcinoma and renal cell carcinoma.^[^ ^60^, ^61^ ^]^ Additionally, we found that the promotion of stemness and proliferation of GSCs induced by VRK1 overexpression can be inhibited by *YBX1* knockdown, indicating that VRK1 regulates the stemness and proliferation of GSCs via YBX1. We propose that the VRK1/YBX1/SOX2 pathway regulates the stemness and proliferation of GSCs. In clinical tissue specimens, VRK1, YBX1, and SOX2 were significantly overexpressed in glioma, with expression levels increasing with pathological grade, but were weakly expressed in non‐tumor tissues. Correlation analysis revealed a positive correlation among VRK1, YBX1, and SOX2 at the protein level in glioma tissues, further supporting the regulatory relationship among VRK1, YBX1, and SOX2. In GBM patients with high VRK1 expression, YBX1 and SOX2 were also overexpressed, suggesting that GSCs in these patients are highly proliferative and more likely to exhibit treatment resistance and tumor recurrence. Therefore, targeting the VRK1/YBX1/SOX2 axis may offer a promising therapeutic strategy for glioma treatment.

Small‐interfering RNA (siRNA)‐encapsulated nanoparticle platform represents a transformative advancement in next‐generation therapeutics for central nervous system diseases.^[^ ^62^ ^]^ Leveraging recent breakthroughs in nanomedicine, this drug delivery system enables the synergistic co‐delivery of therapeutic payloads with enhanced target specificity, thereby facilitating precision oncology applications. Given the lack of effective inhibitors targeting VRK1,^[^ ^63^ ^]^ we engineered A/TMZ‐siVRK1, a VRK1‐targeting nanoliposome that co‐delivers siRNA against VRK1 with TMZ. This innovative combination aims to enhance therapeutic efficacy by simultaneously targeting VRK1 and delivering TMZ directly to tumor cells, establishing a novel combinatorial therapeutic strategy for GBM. Our research demonstrated that A/TMZ‐siVRK1 effectively targeted glioma tissues, inhibited tumor proliferation, and prolonged survival time in an intracranial tumor xenograft murine model. Mechanistically, nanoliposome‐mediated delivery of siVRK1 significantly suppressed the VRK1/YBX1/SOX2 signaling pathway, which is crucial for maintaining the stemness and proliferation of GSCs. By disrupting this pathway, A/TMZ‐siVRK1 not only inhibited tumor growth but also enhanced the sensitivity of glioma cells to TMZ, thereby improving overall treatment outcomes. A/TMZ‐siVRK1 represents a novel and effective combinatorial therapeutic strategy for GBM. In the future, the combination of molecular targeted drugs and histone epigenetic enzyme inhibitors delivered via nanoliposomes holds great promise for providing a more effective therapeutic strategy.

In conclusion, this study establishes a link between the metabolite lactate in the tumor microenvironment and the stemness regulation of GSCs. Lactate regulates the stemness and proliferation of GSCs via VRK1 in GBM, providing a novel theoretical basis for understanding GBM recurrence and treatment resistance. Furthermore, lactate promotes VRK1 expression by inducing histone lactylation at H3K18, thereby regulating the stemness and proliferation of GSCs. This finding provides new evidence that histone lactylation drives tumor progression by modulating gene expression. Finally, the VRK1/YBX1/SOX2 pathway regulates the stemness and proliferation of GSCs, and the VRK1‐targeted nanoliposome A/TMZ‐siVRK1 effectively inhibits the stemness and proliferation of GSCs, highlighting its therapeutic potential in GBM (**Figure** **11**).

**Figure 11:** Schematic illustration (authorized by BioRender) of lactate regulates the stemness and proliferation of glioma stem cells via H3K18la/VRK1/YBX1/SOX2.

## 4 Experimental Section

### Ethics Statement and Human Specimens

All animal experiments in this study were conducted in accordance with the guidelines of the China Medical University Animal Care and Use Committee and were approved by the Ethics Committee of China Medical University (Approval No. CMU20240701). The human glioma tissue samples used in this study were collected from the First Hospital of China Medical University and Shengjing Hospital of China Medical University (Table S2, Supporting Information), which was approved by the Ethics Committee of the First Hospital of China Medical University (Approval No. KLS202286) and Shengjing Hospital of China Medical University (Approval No. 2024PS107K). Histopathological diagnoses were independently confirmed by two neuropathologists according to the WHO classification guideline. All samples were de‐identified before being processed.

### Dataset Preparation and Gene Screening Process

RNA sequencing (RNA‐seq) data and corresponding clinical information from the TCGA dataset were obtained from the GlioVis website (http://recur.bioinfo.cnio.es/), including 625 samples (Grade II glioma: 227 cases, Grade III glioma: 243 cases, GBM: 155 cases).^[^ ^64^ ^]^ RNA‐seq data and associated clinical data from the CGGA dataset were downloaded from the CGGA website (http://www.cgga.org.cn), including 309 samples (Grade II glioma: 105 cases, Grade III glioma: 67 cases, GBM: 137 cases). RNA‐seq data from the GSE145699 dataset and GSE67089 dataset were retrieved from the Gene Expression Omnibus (GEO) database. The GSE145699 dataset includes 12 sequencing profiles derived from three GBM cell lines, both with and without lactate treatment. The GSE67089 dataset comprises 10 DGC samples and 30 GSC samples.

### Cell Model Construction

GSCs used in this study were derived from four clinical GBM tissue specimens.^[^ ^37^, ^38^ ^]^ CD133‐positive cells were isolated from primary cells derived from GBM specimens using magnetic‐activated cell sorting (MACS), followed by short tandem repeat (STR) analysis for authentication. Western blot was performed to assess the expression of stemness markers, including SOX2, SOX9, OLIG2, CD133, NES, and POU3F2. CD133 expression was further confirmed by immunofluorescence staining. Additionally, in vivo tumorigenicity assays were performed to evaluate the tumor‐forming capacity of GSCs. Cells exhibiting stem cell characteristics, as confirmed by the above detection, were designated as GSCs, named GSC4, GSC21, GSC40, and GSC63, respectively.

### Cell Culture and Cell Transfection

Primary patient‐derived glioma stem cells (GSC4, GSC21, GSC40, and GSC63) and their corresponding differentiated glioma cells (PGC4, PGC21, PGC40, and PGC63) were derived from fresh GBM tissues immediately after surgery at the First Hospital of China Medical University.^[^ ^37^ ^]^ DGCs were cultured in RPMI‐1640 medium supplemented with 10% FBS and 1% penicillin/streptomycin at 37 °C with 5% CO_2_. GSCs were cultured in Dulbecco's Modified Eagle's Medium/Nutrient F‐12 (DMEM/F12) supplemented with 2% B27, 20 ng/mL epidermal growth factor (EGF), 20 ng/mL basic fibroblast growth factor (bFGF), and 1% penicillin/streptomycin at 37 °C with 5% CO_2_.^[^ ^37^ ^]^ HEK293T cells were cultured in high‐glucose DMEM media supplemented with 10% FBS and 1% penicillin/streptomycin at 37 °C with 5% CO_2_.

Lentivirus vectors for *VRK1* knockdown (shVRK1) and *VRK1* overexpression were obtained from GeneChem. Lentiviral transduction was performed as previously described.^[^ ^37^ ^]^ The shRNA sequences used were as follows: shVRK1‐1, GAAGTAAGGATGATGGCAAAT; shVRK1‐2, GTAGATTATGGCCTTGCTTAT. Cells were transfected with lentiviral particles according to the manufacturer's instructions. After transduction with the shRNA constructs, stable cell lines were selected using 5 µg/mL puromycin solution.

### Extreme Limiting Dilution Analysis (ELDA)

The neurosphere‐forming and self‐renewal capabilities of GSCs were evaluated using the ELDA web‐based tool. The cells were dissociated with Accutase and seeded into 96‐well plates at densities of 1, 10, 25, 50, 100, and 250 cells per well. After 7 days of culture, the number of neurospheres with diameters exceeding 60 µm was counted in each well. Data were subsequently analyzed using the ELDA tool available at https://bioinf.wehi.edu.au/software/elda/.

### Neurosphere Formation Assay

The neurosphere‐forming capability of GSCs was assessed by the number of neurospheres formed. The cells were dissociated with Accutase and seeded into 24‐well plates at a density of 1000 cells per well. After 7 days of culture, the number of neurospheres with diameters exceeding 60 µm was counted in a single field of view.

### Neurosphere Proliferation Assay

The proliferative capability of GSCs was evaluated by the size of the neurospheres formed. The cells were seeded into 96‐well plates at a density of 1000 cells per well. After 7 days of culture, the diameter of individual neurospheres was measured in a representative microscopic field.

### In Vivo Limiting Dilution Assay

Lentivirus vectors were used to establish stable *VRK1*‐knockdown GSC63 cell lines (shVRK1‐1 and shVRK1‐2) and a control cell line (NC). NC, shVRK1‐1, and shVRK1‐2 cells were prepared at various cell doses (10, 100, 1000, and 10 000 cells) and intracranially injected into 6‐week‐old BALB/c nude mice (*n* = 5). On day 30, the mice were euthanized, and brain tissues were collected for H&E staining to assess the tumor formation rate. Statistical analysis was performed using the ELDA tool available at https://bioinf.wehi.edu.au/software/elda/.

### Intracranial Tumor Xenograft Transplantation

Six‐week‐old male nude mice were raised in laminar flow cabinets under specific pathogen‐free (SPF) conditions at the Laboratory Animal Center of China Medical University. Mice were anesthetized with isoflurane and positioned in a stereotactic frame. GSC63 cell suspension (2 × 10^4^ cells in 2 µL) was injected into the right cerebral hemisphere at a depth of 2.5 mm, 2 mm to lateral to the sagittal suture, and 2 mm posterior to the coronal suture. The injection was performed at a rate of 0.5 µL/min for 4 min. Mice were monitored daily and euthanized when they exhibited neurological symptoms or experienced a weight loss exceeding 20%. Survival time was recorded and compared among different experimental groups. Additionally, at a predetermined time point, a separate cohort of mice from each group was euthanized to collect brain tissues for further histological analysis.

### Real‐Time Quantitative PCR (RT‐PCR)

Total RNA was extracted using TRIzol reagent (Invitrogen) according to the manufacturer's instructions. Subsequently, RNA was reverse‐transcribed into cDNA using PrimeScript RT Master Mix (TaKaRa). RT‒qPCR was performed on a thermal cycler (Roche) using SYBR Green Master Mix (TaKaRa). The thermal cycling conditions were as follows: 1 cycle of 95 °C for 30 s, followed by 40 cycles of a two‐step cycling program (95 °C for 5 s, 60 °C for 30 s). The relative mRNA expression levels of target genes were calculated using the 2^‐^ΔΔCt method and normalized to *18S* rRNA expression. The PCR primer sequences were provided in Table S3 (Supporting Information).

### Western Blot

Total proteins were extracted using RIPA lysis buffer supplemented with protease inhibitor and phosphatase inhibitor. Protein concentrations were determined using a Bicinchoninic Acid (BCA) Assay Kit (Beyotime). The protein extracts were separated by sodium dodecyl sulfate‐polyacrylamide gel electrophoresis (SDS‐PAGE) and subsequently transferred onto polyvinylidene fluoride PVDF membranes (Cytiva). The protein‐containing membranes were blocked with 5% skim milk at room temperature for 1 h, followed by overnight incubation with primary antibodies at 4 °C. Afterward, the membranes were incubated with secondary antibodies at room temperature for 1 h. Protein bands were visualized using the enhanced chemiluminescence (ECL) substrate (Tanon). The antibodies used in this study were listed in Table S4 (Supporting Information).

### Immunofluorescence Staining

Cells were dissociated into single‐cell suspensions using Accutase and seeded onto confocal dishes pre‐coated with 0.5% laminin. After adherence, cells were fixed with methanol for 15 min and permeabilized with 0.5% Triton X‐100 for 20 min. Following blocking with 5% bovine serum albumin (BSA) for 1 h at room temperature, cells were incubated with anti‐YBX1 primary antibody at 4 °C overnight. Subsequently, the samples were incubated with Multi‐rAb™ CoraLite® Plus 594‐conjugated secondary antibody and counterstained with DAPI. The stained samples were imaged using a confocal fluorescence microscope.

### Immunohistochemistry (IHC)

Paraffin‐embedded tissue specimens were sectioned at 4‐µm thickness. H&E staining was performed according to standard protocols. For IHC, the streptavidin‐biotin immunostaining method was employed. Tumor sections were deparaffinized in xylene, rehydrated through graded ethanol solutions, subjected to antigen retrieval, blocked with blocking agent, and incubated with primary antibodies overnight at 4 °C. The primary antibodies used were: anti‐VRK1 antibody (1:100, Abcam), anti‐YBX1 antibody (1:200, Proteintech), anti‐SOX2 antibody (1:200, Proteintech), and anti‐Ki67 antibody (1:2000, Proteintech). On the following day, the sections were incubated with secondary antibodies, followed by DAB staining, hematoxylin counterstaining, hydrochloric acid acidification, and dehydration. The staining intensity of each tissue section was evaluated at 400× magnification in five randomly selected fields of view. The expression levels of VRK1, YBX1, and SOX2 were assessed based on staining intensity and distribution using the immunoreactive score (IRS), calculated as: IRS = staining intensity (SI) × percentage of positive cells (PP). SI was scored as: 0 (absent), 1 (weak), 2 (moderate), 3 (strong). PP was scored as: 0 (0%), 1 (1%–25%), 2 (26%–50%), 3 (51%–75%), 4 (76%–100%).^[^ ^37^ ^]^

### Chromatin Immunoprecipitation (ChIP)

ChIP assays were performed using the SimpleChIP Enzymatic Chromatin IP Kit (Cell Signaling Technology) according to the manufacturer's protocol. Immunoprecipitation reactions were conducted using 5 µg of anti‐H3K18la antibody (PTM BIO) and anti‐YBX1 antibody (1:20, Proteintech), with normal IgG serving as a negative control. Purified DNA was subjected to qPCR analysis using primers targeting the *VRK1* and *SOX2* promoter region. Relative chromatin enrichment was calculated as the amount of amplified DNA, normalized to input and relative to values obtained after normal IgG immunoprecipitation.

### Immunoprecipitation Mass Spectrometry (IP‐MS)

VRK1 immunoprecipitates and corresponding control IgG immunoprecipitates prepared from GSC63 cell lysates were resolved on SDS‐PAGE gels. Protein bands were excised from the gels and subjected to LC‐MS/MS analysis. Swissprot_Human mass spectra were used as the standard reference. Trypsin/P was used for cleavage. Mass spectrometry data were captured and analyzed by Beijing Novogene Technology Company.

### In Vitro Kinase Assay

Recombinant human VRK1 and YBX1 proteins were purchased from Abcam. The kinase activity of VRK1 was measured using a non‐radioactive method with an anti‐phospho‐serine antibody (Life Technologies). Kinase reactions were performed in a total volume of 20 µL, containing 100 ng of YBX1, variable amounts of recombinant kinase VRK1 (100, 200, and 500 ng), and 100 µm ATP in kinase buffer (Cell Signaling Technology) at 30 °C for 30 min. The reactions were terminated by adding 10 mm EDTA and stored at −20 °C until analysis by immunoblotting. Coomassie brilliant blue staining was used to visualize YBX1 and VRK1 proteins.

### Co‐Immunoprecipitation (Co‐IP)

Cells were collected and lysed in 400 µL of lysis buffer supplemented with protease inhibitor for 30 min on ice. After centrifugation, the supernatant was collected and incubated with 2 µg of primary antibody (anti‐VRK1, anti‐YBX1, or anti‐SOX2) or control IgG at 4 °C overnight. Subsequently, 50 µL of protein A/G magnetic beads were added and incubated for 2 h at room temperature. The binding complexes were collected, washed three times with washing buffer, and eluted by boiling in loading buffer. The samples were analyzed by western blotting.

### Glutathione S‐Transferase (GST) Pull‐Down Assay

GST‐labeled VRK1 wild‐type purified protein (VRK1 WT) and GST‐labeled VRK1 K71 mutant purified protein (VRK1 K71M) were constructed by OBiO Technology. GST‐labeled VRK1 purified protein (VRK1 WT or VRK1 K71M) was incubated with recombinant YBX1 protein (Abcam) at 4 °C overnight. After incubation, protein complexes were captured using GST magnetic beads, washed three times to remove non‐specific binding, and eluted by boiling in loading buffer. The eluted proteins were then analyzed by immunoblotting.

### Ubiquitination Assay

Cells transfected with *VRK1* knockdown, *VRK1* overexpression, or control vectors were treated with 10 µm MG132 for 6 h prior to lysis. A total of 1 mg of protein was subjected to co‐immunoprecipitation. YBX1 was pulled down using an anti‐YBX1 antibody at 4 °C overnight. The level of YBX1 ubiquitination was assessed by western blot using an anti‐Ub antibody.^[^ ^65^ ^]^

### Preparation and Characterization of A/TMZ‐siVRK1, A/TMZ‐siNC, and A/PLGA‐ siVRK1

Preparation of A/TMZ‐siVRK1 via a single‐step nanoprecipitation method. TMZ, cholesterol, PEG_2000_‐DSPE, and Angiopep‐2‐PEG_2000_‐DSPE were dissolved in 200 µL of DMSO. The mixture of TMZ/PEG_2000_‐DSPE/Angiopep‐2‐PEG_2000_‐DSPE (mass ratio of 30:20:1) was vortexed for 5 min and stirred at room temperature for 3 h. DOTAP was dissolved in DMSO at a concentration of 50 mg/mL and combined with siVRK1 at an N:P ratio of 10:1 in 800 µL of DEPC water, followed by stirring for 1 h. The TMZ/PEG_2000_‐DSPE/Angiopep‐2‐PEG_2000_‐DSPE mixture was slowly dripped into water to form A/TMZ‐siVRK1 nanoparticles. Due to their amphiphilic nature, PEG_2000_‐DSPE, Angiopep‐2‐PEG_2000_‐DSPE, and cholesterol self‐assemble at the water‐oil interface, with hydrophilic head groups oriented toward the aqueous phase and hydrophobic tails embedded within the hydrophobic TMZ aggregates. Subsequently, dialysis was performed to remove DMSO from the A/TMZ‐siVRK1 solution. A/TMZ‐siVRK1 was concentrated using an Amicon Ultra‐4 centrifugal filter (Millipore) with a molecular weight cutoff of 10000 Da. Similarly, A/TMZ‐siNC was prepared by replacing siVRK1 with an equivalent amount of negative control siRNA (siNC). A/PLGA‐siVRK1 was obtained by substituting TMZ with an equivalent mass of PLGA. The siVRK1 sequence targets the 5′‐GAAGUAAGGAUGAUGGCAAAU‐3′ region, with the empty vector used as a negative control.

Particle size, zeta potential, and stability in serum (10%) were determined using a Zetasizer Nano‐ZS90 (Malvern, UK). Morphology was observed using a Tecnai G2 Spirit Twin transmission electron microscope (FEI, USA). Samples dispersed in PBS were dropped onto a 200‐mesh copper grid before recording TEM images.

Drug loading (DL) and encapsulation efficiency (EE) of TMZ were analyzed using ultra‐performance liquid chromatography‐tandem mass spectrometry (UPLC‐MS/MS). The chromatographic column was an Agilent TC‐C18 with dimensions 150 × 4.6 mm, and the mobile phase was a mixture of water containing 0.1% formic acid and methanol containing 0.1% formic acid (7:3) at a flow rate of 0.4 mL/min. Mass spectrometer parameters were as follows: Capillary, 3.5 kV; Cone, 66 V; Collision, 32 V; Ion source temperature, 250 °C; Desolvation Gas Flow, 11 L/min; Cone Gas Flow, 7 L/min; m/z: 195.0‐138.2. The prepared A/TMZ‐siVRK1 nano‐prodrugs were lyophilized to obtain dry powder A/TMZ‐siVRK1 nano‐prodrugs. The lyophilized nano‐prodrug powder was dissolved in 1 mL of water containing 0.1% formic acid, and an equal volume of methanol containing 0.1% formic acid was added. The samples were measured in triplicate at 10 µL per injection. The prepared A/TMZ‐siVRK1 nano‐prodrug solution was transferred to a dialysis bag and dialyzed for 6 h to remove free TMZ. The concentration of TMZ in the solution within the dialysis bag was then measured to detect the encapsulation efficiency. A standard curve was prepared with TMZ aqueous solutions ranging from 0 to 100 µg/mL, and the concentration was determined.

(1) $$Y=0.113151\times X+0.889779,\;\;R^{2}=0.992$$

(2) $$\mathrm{EE}\left(\%\right)=\left(\mathrm{weight}\;\mathrm{of}\;\mathrm{drug}\;\mathrm{loaded}\right)/\left(\mathrm{weight}\;\mathrm{of}\;\mathrm{drug}\;\mathrm{in}\;\mathrm{feed}\right)\times 100\%$$

(3) $$\begin{array}{c} \mathrm{DL}\left(\%\right)=\left(\mathrm{weight}\;\mathrm{of}\;\mathrm{drug}\;\mathrm{loaded}\right)/\left(\mathrm{weight}\;\mathrm{of}\;\mathrm{nanoliposomes}\right)\times 100\% \end{array}$$

(4) $$\mathrm{EE}\left(\%\right)\mathrm{of}\;\mathrm{TMZ}=72.54\%\pm 2.63\%$$

(5) $$\mathrm{DL}\left(\%\right)\mathrm{of}\;\mathrm{TMZ}\;\mathrm{in}\;A/\mathrm{TMZ}-\mathrm{siVRK}1=37.45\%\pm 2.83\%$$

### Drug Release

1 mL A/TMZ‐siVRK1 nanoliposomes were transferred into a dialysis bag with a molecular weight cutoff of 3500 Da and then immersed in 50 mL of PBS at pH 7.4 or pH 6.5, respectively. Drug release was monitored at 37 °C. At various time points, 500 µL of the sample was withdrawn and stored at 4 °C, while an equivalent volume of PBS was added to maintain a constant volume. The released TMZ and si‐VRK1 were detected using UPLC‐MS/MS and a fluorescence microplate reader, respectively. The detection method and mass spectrometry conditions for TMZ were the same as described.^[^ ^62^ ^]^ siVRK1 was conjugated with FITC following the preparation method described to produce A/TMZ‐siVRK1‐FITC. At different time points, 500 µL of the sample was withdrawn and stored at 4 °C, while an equivalent volume of PBS was added to maintain a constant volume. The samples were transferred to a 96‐well plate, avoiding light exposure. The fluorescence intensity of FITC was measured using a microplate reader to calculate the release efficiency of siVRK1.

### Endosomal Escape of A/TMZ‐siVRK1

GSC63 cells were dissociated into single cells using Accutase, then seeded into 6‐well plates pre‐coated with 0.5% laminin. A/TMZ‐siVRK1‐FITC nanoliposomes were added to the wells and incubated for 1, 4, and 8 h, respectively. After washing twice with PBS, cells were incubated in DMEM/F12 medium containing Lysotracker‐Red for 30 min. Subsequently, cells were collected for confocal laser scanning microscopy (CLSM) analysis. Fluorescence colocalization analysis was performed using ImageJ software (version 2.9.0).

### Detection of A/TMZ‐siVRK1 Penetrating the Blood‐Brain Barrier

GSC63 cells were dissociated with Accutase and seeded on the lower chamber of the Transwell system pre‐coated with 0.5% laminin. HBMEC cells were cultured in the upper chamber of the Transwell. Blood‐brain barrier integrity was confirmed when transendothelial electrical resistance (TEER) reached 200 Ω•cm^2^. A/TMZ‐siVRK1‐FITC and TMZ‐siVRK1‐FITC nanoliposomes were added to the upper chamber of the Transwell. After 4 h of incubation, the fluorescence intensity of FITC in HBMEC and GSC63 cells incubated with A/TMZ‐siVRK1/FITC was detected using confocal laser scanning microscopy. The cell membrane of HBMEC was labeled with the DIO fluorescence dye, while the nucleus of GSC63 was stained with DAPI. After incubation for 4 h, the fluorescence intensity of the upper and lower chambers was measured using a microplate reader. The proportion of A/TMZ‐siVRK1/FITC and TMZ‐siVRK1/FITC penetrating the blood‐brain barrier was determined by calculating the ratio of the fluorescence intensity in the lower chamber to the sum of the fluorescence intensity in the upper and lower chambers. The calculation formula is as follows:

(6) $$\begin{array}{ccc} \mathrm{Penetration}\;\mathrm{rate}\;\left(\%\right) & = & \left(\mathrm{Fluorescence}\;\mathrm{intensity}\;\mathrm{in}\;\mathrm{the}\;\mathrm{upper}\;\mathrm{chamber}\right)\\ & & /\left(\mathrm{Fluorescence}\;\mathrm{intensity}\;\mathrm{in}\;\mathrm{the}\;\mathrm{upper}\;\mathrm{chamber}\;\right.\\ & & +\left.\mathrm{Fluorescence}\;\mathrm{intensity}\;\mathrm{in}\;\mathrm{the}\;\mathrm{lower}\;\mathrm{chamber}\right)\\ & & \;\;\times \;100\%. \end{array}$$

### Pharmacokinetic Testing

An orthotopic xenograft tumor model was established in nude mice using GSC63 cells. TMZ, siVRK1‐FITC, and A/TMZ‐siVRK1‐FITC were administered via tail vein injection (the equivalent dose of TMZ and siVRK1 was 30 and 0.5 mg/kg). At various time points (5, 10, 20, and 30 min, 1, 2, 4, 8, 12, and 24 h), 100 µL of blood collected from the tail vein, 1 mg of GBM tissue, and normal brain tissue were transferred into medical anticoagulant tubes, respectively. Then, 10 µL of 10% phosphoric acid was added, and the samples were centrifuged at 15 000 rpm. 50 µL of plasma was aspirated and transferred to new 1.5 mL centrifuge tubes. An additional 50 µL of protein precipitation agent (a mixture of acetonitrile and 10% trichloroacetic acid in a 2:3 ratio) was added. The plasma was thoroughly mixed and centrifuged again at 15 000 rpm for 10 min. The supernatant was aspirated using a pipette, filtered, and then 1 µL was injected. The concentration of TMZ in each tissue was determined using UPLC‐MS/MS. The fluorescence intensity of siVRK1‐FITC in each group was detected by a microplate reader.

### In Vivo Tissue Targeting Distribution Analysis and Detection of Drug Content in Brain Tissue

A/TMZ‐siVRK1‐Cy5 and TMZ‐siVRK1‐Cy5 were injected into mice via the tail vein. After 24 h, the mice's major organs were dissected out and imaged by a small animal imaging system. TMZ, siVRK1‐FITC, and A/TMZ‐siVRK1‐FITC were injected into tumor‐bearing mice via the tail vein. Mice were euthanized at the 6 and 12th hours after administration. Tumor tissues were removed, weighed, placed in plastic tubes, and 1 mL of PBS containing 1% phosphoric acid was added and homogenized with a high‐speed shear machine. Then, 300 µL homogenate sample was previously taken and placed in a 1.5 mL centrifuge tube, 300 µL protein precipitant (10% trichloroacetic acid: acetonitrile = 3:2) was added, vortexed for 30 s, and centrifuged at 12 000 rpm for 10 min. The supernatant was filtered, and the concentration of TMZ in tumor tissues of each group was determined using the same methods. The fluorescence intensity of siVRK1‐FITC was detected using a microplate reader.

### Statistical Analysis

Statistical analyses were performed using GraphPad Prism 9.0 and R 4.0.3 software. The statistical differences of data were analyzed with the unpaired two‐tailed Student's t test for two‐group comparison and one‐way analysis of variance (ANOVA) for multiple‐group comparison. Pearson correlation analysis was used to calculate the correlation between variables. Data were presented as mean ± standard deviation of measurement (SD). A value of *p* < 0.05 was considered statistically significant: ^*^ *p* < 0.05, ^**^ *p* < 0.01, ^***^ *p* < 0.001, ^****^ *p* < 0.0001. *p* > 0.05 indicated no significant difference and was marked with ns.

## Conflict of Interest

The authors declare no conflict of interest.

## Author Contributions

J.L. and Q.G. conceived the project. J.L., Q.G., X.Z., and R.X. designed the project. Q.G., J.L., X.Z., R.X., and C.T. performed experiments. J.L., Q.G., and X.Z. analyzed the data. J.L. and Q.G. wrote the manuscript. Q.G., R.X., and X.Z. supervised the project. All authors read and approved the final version of the manuscript.

## Supporting information



Supporting Information

## Data Availability

The data that support the findings of this study are available from the corresponding author upon reasonable request.
